The article "Diabetes Risk Data Mining Method Based on Electronic Medical Record Analysis" was retracted in 2023. Reasons: unreliable results or conclusions; concerns about the data; concerns about the peer review; concerns about the citations.

# Diabetes Risk Data Mining Method Based on Electronic Medical Record Analysis

**DOI:** 10.1155/2021/6678526

**Published:** 2021-03-04

**Authors:** Yang Liu, Zhaoxiang Yu, Yunlong Yang

**Affiliations:** ^1^Department of Endocrine, Affiliated Hospital of Beihua University, Jilin 132012, China; ^2^Department of Anesthesiology, Affiliated Hospital of Beihua University, Jilin 132012, China; ^3^Department of Cardiothoracic Vascular Surgery, Affiliated Hospital of Beihua University, Jilin 132012, China

## Abstract

In today's society, the development of information technology is very rapid, and the transmission and sharing of information has become a development trend. The results of data analysis and research are gradually applied to various fields of social development, structured analysis, and research. Data mining of electronic medical records in the medical field is gradually valued by researchers and has become a major work in the medical field. In the course of clinical treatment, electronic medical records are edited, including all personal health and treatment information. This paper mainly introduces the research of diabetes risk data mining method based on electronic medical record analysis and intends to provide some ideas and directions for the research of diabetes risk data mining method. This paper proposes a research strategy of diabetes risk data mining method based on electronic medical record analysis, including data mining and classification rule mining based on electronic medical record analysis, which are used in the research experiment of diabetes risk data mining method based on electronic medical record analysis. The experimental results in this paper show that the average prediction accuracy of the decision tree is 91.21%, and the results of the training set and the test set are similar, indicating that there is no overfitting of the training set.

## 1. Introduction

Diabetes is a group of endocrine and metabolic diseases caused by absolute or relative lack of insulin in the human body [1]. Its main feature is increased blood glucose (blood sugar) levels. It is currently one of the most important chronic noncommunicable diseases in the world. Approximately 425 million people worldwide suffer from diabetes. The number of diabetic patients in my country ranks first in the world, and the incidence of diabetes and its related complications is gradually showing an explosive growth, which greatly affects the quality of life of residents and threatens the healthcare system of the entire society [2].

Electronic medical records are the sum of clinical information, visits and observations, diagnosis and treatment plans, pathological explanations, medical measures, and results. In China, the generalization of electronic medical records mainly focuses on the process of medical staff's diagnosis and treatment activities. The medical records of various data such as texts, tables, images, and images generated during the individual's medical treatment are integrated and detailed [3]. As an information carrier for a large number of patients' long-term health information, disease status, diagnosis information, and other data, electronic medical records are massive, high-dimensional, discrete data, which contain a wealth of knowledge. The electronic medical record digitizes the patient's treatment and health status, so that data mining technology can be used to dig out the available pattern features and implicit knowledge. We can use electronic medical record data mining to predict the disease risk of patients and then conduct early intervention for high-risk patients to reduce or reduce the risk of chronic diseases, which can further reduce the incidence of diabetes in the population [1].

The article "Diabetes Risk Data Mining Method Based on Electronic Medical Record Analysis" was retracted in 2023. Reasons: unreliable results or conclusions; concerns about the data; concerns about the peer review; concerns about the citations.

Lovelace S uses a phased, iterative, and participatory approach to improve healthcare, which requires time and resources to carry out the work. Particularly for professionals, the reality is that constraints related to human resources, cost, and time may affect the rigor of data collection and analysis. In this case, the project team may rely on tacit knowledge and expertise to fill in potential gaps in understanding and verifying design decisions. Lovelace S's research team analyzed this problem by using computer-aided qualitative data analysis software and qualitative research coding methods, which are video data samples collected from a series of electronic medical record workflow simulations originally used to support the implementation of electronic medical records. In the context of design, development, and implementation, the comparison and discussion of video analysis methods and corresponding costs are compared and discussed. This study lacks case evidence and is weak in persuasiveness [4]. The Donazar-Ezcurra M study found that identifying people at risk for type 2 diabetes and gestational diabetes is essential to implement preventive interventions to deal with these common diseases. Dietary-Based Diabetes Risk Score is a simple score based only on dietary components and shows a strong inverse correlation with type 2 diabetes events. The purpose of Donazar-Ezcurra M was to assess the association between diet-based diabetes risk scores and gestational diabetes risk in a group of Spanish university graduates. The experiment included data on 3455 women who notified pregnancy between 1999 and 2012. The development of a diet-based diabetes risk score in the study aims to quantify the association between adherence to the prior diet score and the incidence of type 2 diabetes,; among the 9 food categories for which diet scores (reported to be negatively correlated with the incidence of type 2 diabetes), 3 food categories are reported to be directly related to type 2 diabetes. Donazar-Ezcurra M assessed three types of compliance with diet-based diabetes risk scores: low (11–24), intermediate (25–39), and high (40–60). Compared with the lowest category, the higher category showed an independent inverse correlation with the risk of developing gestational diabetes (multivariate-adjusted OR 0·48; 95% CI 0·24, 0·99; linear trend P: 0·01). This research may be one-sided and not practical [5]. Lu H believes that classification is one of the data mining problems that have attracted widespread attention in the database community recently. He proposed a method of using neural networks to discover symbol classification rules. Prior to this, neural networks have not been considered suitable for the privacy protection data sharing hybrid method in the data mining environment, because there is no clear definition of how to classify as a symbolic rule suitable for human verification or interpretation [2]. Lu H believes that the proposed method can extract high-precision concise symbolic rules from the neural network; for example, first train the network to achieve the required accuracy; then, delete the redundant connections of the network through the network pruning algorithm; analyze the activation values of hidden units in the network; use the analysis results to generate classification rules; finally, Lu H's experimental results for a set of standard data mining test problems clearly prove the effectiveness of the method [6]. This research method is highly innovative but complicated to operate and is not suitable for popularization in practical applications [7].

The article "Diabetes Risk Data Mining Method Based on Electronic Medical Record Analysis" was retracted in 2023. Reasons: unreliable results or conclusions; concerns about the data; concerns about the peer review; concerns about the citations.

The innovations of this paper are as follows: (1) proposing the use of decision tree algorithm for data mining of diabetes risk based on electronic medical record analysis; (2) proposing the use of random forest algorithm for data mining of diabetes risk based on electronic medical record analysis; (3) designing a diabetes risk data mining system based on electronic medical record analysis.

## 2. Strategy of Diabetes Risk Data Mining Method Based on Electronic Medical Record Analysis

### 2.1. Data Mining Based on Analysis of Electronic Medical Records

#### 2.1.1. Data Preprocessing of Electronic Medical Records

The “noise” processing of the electronic medical record data is the process of removing irrelevant data in the electronic medical record and retaining useful data.

Carry out content screening processing on the sorted electronic medical record data [8]. According to the different research purposes, different medical records in the electronic medical records are selected, and different attribute information in the medical records is screened according to different target attributes. After data selection, the research data is determined [9].

The standardized adjustment of the electronic medical record text data includes the sorting of input data, the processing of missing data, and the correction of error information. The data protocol is to make the data more standardized and easier to process on the basis of being close to the original data [10]. This stage is to standardize the data after cleaning and selection [11].

#### 2.1.2. Data Mining of Electronic Medical Records

With the rapid growth of medical record data in electronic medical record databases, how to find valuable information or knowledge from a large amount of data has become a hot topic in the research of electronic medical record systems [12]. Electronic medical record data mining is a new research field used for production and development to meet the above needs. It can explore the hidden rules and standards of medical diagnosis in the electronic medical record system and provide assistant decision-making for physicians in the diagnosis and treatment of diseases [13].

The data object of the electronic medical record mining operation is the data in the electronic medical record database. The data in the electronic medical record database is very rich, including patient personal data, medical record data, disease course data, various laboratory examination data, and discharge data. It has the following main characteristics: diversity, incompleteness, and dynamics. Aiming at such data characteristics, we must design a structured electronic medical record. Only in this way, the data in the electronic medical record database can be mined with data mining technology [14, 15].

Export relevant medical information to the electronic medical record database, and mine the hidden medical diagnosis rules and standards in order to provide scientific and accurate auxiliary decision-making for the diagnosis and treatment of diseases [16]. The data collected by the electronic medical record systems of different hospitals is actually patient data, and the amount of data is quite large. From these data sets, different data mining techniques are used to study the relationship between different diseases and the development of different diseases; and to summarize the efficacy of different treatment plans, it has great value for the diagnosis, treatment, and medical research of this disease [17].

The article "Diabetes Risk Data Mining Method Based on Electronic Medical Record Analysis" was retracted in 2023. Reasons: unreliable results or conclusions; concerns about the data; concerns about the peer review; concerns about the citations.

### 2.2. Classification Rule Mining

#### 2.2.1. Decision Tree Algorithm

Among classification data mining algorithms, decision tree algorithm is the most commonly used algorithm. Decision tree algorithm combines the classification process of tree shape and adaptation problem [18]. There is a shared attribute in the specified tree; that is, each layer corresponds to a classification attribute. The nodes in the layer have different attribute values, and the corresponding data of the attribute values are stored in the nodes [19]. Each node stores the probability distribution of different types of label attributes on the branch line [20].

Assume that the current node is V, the training data set that reaches V is *L*, there are *k* different category labels *C*_*i*_(*i* = 1,2,…, *k*), the tuple set of *L* and category label *C* is *C*_*i*,*L*_, and *C*_*i*_, and *l* is divided into *y* subsets {*L*_1_, *L*_2_,…, *L*_*y*_}[21, 22].

*(1) Information Gain*. The information gain on a certain division attribute N is defined as the difference between the amount of information (entropy) needed to identify tuples before division and the amount of information needed to identify tuples after division on attribute N [23]. Here is the following relationship:

(1) $$\begin{array}{c} \text{InfoGain}\left(N\right)=\text{Info}\left(L\right)-{\text{Info}}_{N}\left(L\right),\\ \text{Info}\left(L\right)=-\sum_{i=1}^{k}p_{i}\log_{2}\left(p_{i}\right),\\ p_{i}=P\left(t\in C_{i}|\forall t\in L\right),\\ {\text{Info}}_{N}\left(D\right)=\sum_{j=1}^{y}\frac{\left|L_{j}\right|}{\left|L\right|}\times \text{Info}\left(L_{j}\right). \end{array}$$

*(2) Gain Rate*. The information gain metric tends to use attribute partitioning with more branches, and the gain rate metric is adopted, which uses the split information value to normalize the information gain [24]. The definition formula of split information is as follows:

(2) $$\begin{array}{c} {\text{SplitInfo}}_{N}=-\sum_{j=1}^{y}\frac{\left|L_{j}\right|}{\left|L\right|}\times \;\log_{2}\left(\frac{\left|L_{j}\right|}{\left|L\right|}\right). \end{array}$$

The gain rate is defined as

(3) $$\begin{array}{c} GainRatio\left(N\right)=\frac{InfoGain\left(N\right)}{SplitInfo\left(N\right)}. \end{array}$$

*(3) Gini Indicator*. The Gini index is the measurement criterion used in the CART algorithm. The Gini index measures the impurity of the data partition or the training tuple set *L* [25]. Its definition formula is

(4) $$\begin{array}{c} \text{Gini}\left(L\right)=1-\sum_{i=1}^{k}p_{i}^{2},\\ p_{i}=p\left(t\in C_{i}|\forall t\in L\right). \end{array}$$

The Gini index considers the binary division of each attribute. Assuming that *L* is divided into *L*_1_ and *L*_1_ for a certain binary division of attribute N on *L*, the Gini index of this division is defined as

(5) $$\begin{array}{c} {\text{Gini}}_{N}\left(L\right)=\frac{\left|L_{1}\right|}{\left|L\right|}\text{Gini}\left(L_{1}\right)+\frac{\left|L_{2}\right|}{\left|L\right|}\text{Gini}\left(L_{2}\right). \end{array}$$

The decrease in impurity due to this division is defined as

(6) $$\begin{array}{c} \Delta \text{Gini}\left(N\right)=\text{Gini}\left(L\right)-{\text{Gini}}_{N}\left(L\right). \end{array}$$

Each time the attribute that can maximize the reduction of impurity is selected as the splitting attribute, this attribute and its split subset (discrete value attribute) or split point (continuous value attribute) together form the splitting criterion [26].

The article "Diabetes Risk Data Mining Method Based on Electronic Medical Record Analysis" was retracted in 2023. Reasons: unreliable results or conclusions; concerns about the data; concerns about the peer review; concerns about the citations.

#### 2.2.2. Random Forest Algorithm

Random forest is an ensemble learning method that can perform classification, regression, and other tasks. Random forest constructs multiple decision trees during training, integrates the results of all decision trees as outputs when predicting votes on the output results in classification, and takes the average of the results as output in regression [27]. Compared with traditional decision trees, random forest can effectively overcome the overfitting problem in the classification process [28]. In classification or regression tasks, random forest can effectively rank the importance of features [29].

Use the depth comparison function to calculate the *x* feature of the given data:

(7) $$\begin{array}{c} f_{\theta }\left(I,x\right)=d_{I}\left(x+\frac{u}{d_{I}\left(x\right)}\right)-d_{I}\left(x+\frac{v}{d_{I}\left(x\right)}\right), \end{array}$$

where *d*_*I*_(*x*) is the depth of the training data *x* of the data set I and the parameter *θ*=(*u*, *v*) is the offset value, giving *d*_*I*_(*x*′) a large normal amount [30]. The comparison with the threshold *γ* is used to determine whether the tree branches to the left or right [31]. At the node *t* of the tree, use the function *p*(*c|I*, *x*) to distinguish and store the feature *c* of the data set [32, 33]. The average distribution of all trees in the forest gives the final classification result; The formula is as follows::

(8) $$\begin{array}{c} p\left(c|I,x\right)=\frac{1}{T}\sum_{t=1}^{T}p_{t}\left(c|I,x\right). \end{array}$$

Each tree must be trained on a different random data set, and a set of split candidate parameters *φ*=(*θ*, *γ*) is randomly selected (*θ* is the feature parameter, and *γ* is the threshold) [34].

Divide instance *Q*={(*I*, *x*)} into two left and right subsets *Q*_*I*_(*φ*) and *Q*_*r*_(*φ*):

(9) $$\begin{array}{c} Q_{I}\left(\varphi \right)=\left\{\left(I,x\right)|f_{\theta }\left(I,x\right)<\gamma \right\},\\ Q_{r}\left(\varphi \right)=Q/Q_{I}\left(\varphi \right). \end{array}$$

Calculate the maximum obtained information given by *φ*:

(10) $$\begin{array}{c} \varphi^{\Delta }=\arg\max_{\varphi }G\left(\varphi \right),\\ G\left(\varphi \right)=H\left(\varphi \right)-\sum_{S\in \left(I,r\right)}\frac{\left|Q_{S}\left(\varphi \right)\right|}{\left|Q\right|}H\left(Q_{S}\left(\varphi \right)\right), \end{array}$$

where H(Q) is the data set feature (*I*, *x*) ∈ *Q* that calculates all *l*_*I*_(*x*) of the normalized histogram. If *G*(*φ*^Δ^) is large enough and the depth of the tree is less than the maximum value, recurse the left and right subsets *Q*_*I*_(*φ*^Δ^) and *Q*_*r*_(*φ*^Δ^)[35, 36].

The article "Diabetes Risk Data Mining Method Based on Electronic Medical Record Analysis" was retracted in 2023. Reasons: unreliable results or conclusions; concerns about the data; concerns about the peer review; concerns about the citations.

The method part of this paper uses the above method to study the data mining method of diabetes risk based on electronic medical record analysis. The specific process is shown in Figure 1.

## 3. Experiment on Data Mining Method of Diabetes Risk Based on Electronic Medical Record Analysis

### 3.1. Designing an Electronic Medical Record Diabetes Risk Data Mining System

#### 3.1.1. Frame Design

From the perspective of the software structure hierarchy, referring to the commonly used three-tier architecture, the overall architecture of the electronic medical record data analysis system can be divided into the basic platform, data layer, logical control layer, and user interaction layer from bottom to top.

The electronic medical record data analysis system designed in this paper mainly includes four levels: the basic platform mainly provides the support of the underlying physical environment platform for the system; the database system prepares good conditions for the data information management of the electronic medical record data; the system logic management layer provides the logic application and realization of the basic four functional modules of the system; the visual interface is the concrete realization of the view layer, which is a convenient operation interface for users. In addition, the system safety standards and normative standards running through these four levels provide safety-related guidelines for system design. According to specific business needs, it is clear that the main modules of the electronic medical record data mining analysis system include data sorting, data retrieval, data analysis, and data visualization.

#### 3.1.2. Database Logic Design

The electronic medical record data analysis system is a comprehensive data management and analysis system based on data statistics and analysis. After getting the entity relationship diagram in the conceptual design stage, it needs to be transformed into a logical structure that matches the data model supported by the actual database. The database selected by this system is the open-source relational database MySQL. According to business requirements and data characteristics, the database has designed a total of 6 core tables, which are user information table, patient basic information table, patient illness table, patient hospitalization status table, patient disease and expense table, and patient-specific expense table.

1. User information table: this table contains user login name, password, name, e-mail, and login status. The primary key is the user's login name.
2. Patient basic information table: this table contains basic information of patients in the case, such as gender, age, marriage, ethnicity, occupation, and blood type, and provides a basis for case retrieval and analysis.
3. Patient disease table: this table is the outpatient diagnosis number of the patient in the stored case. In some cases, there will be more than one disease in the case, so the main diagnosis number 1, the main diagnosis number 2, the main diagnosis number 3, and even the main diagnosis number 4 appear.
4. Patient hospitalization table: this table stores the patient's hospitalization information, including admission time, discharge time, hospitalization days, and times.
5. Patient disease and expense table: this table stores the patient's expense status and related diseases. There are mainly total expenses and self-expenses as well as reimbursement expenses, disease types, and diseases.
6. Patient-specific expenditure table: this table describes the personal expenditure information and the destination of the expenditure of the patient in the case.

The article "Diabetes Risk Data Mining Method Based on Electronic Medical Record Analysis" was retracted in 2023. Reasons: unreliable results or conclusions; concerns about the data; concerns about the peer review; concerns about the citations.

### 3.2. System Platform Selection

#### 3.2.1. System Structure

*(1) C/S Structure*. C/S mode is also called client/server mode. Servers usually use high-performance computers, workstations, or small computers and use large-scale database systems, such as Oracle, Sybase, Informix, or SQL servers. Customers must install specific client software. The system operation in C/S mode is completed by the client and server, respectively. By reasonably outsourcing the work to the client and server, making full use of the benefits of the material environment, the overall communication cost of the system is reduced at both ends. The server has the functions of data collection, control, and communication with the client. The server program is responsible for the effective management of system resources; the client includes communication with the server and the user interface unit.

*(2) B/S Structure*. B/S is the abbreviation of browser/server. Only browser programs such as Netscape Navigator or Internet Explorer should be installed on the client computer. The server is installed with databases such as Oracle, Sybase, Informix, or SQL server, and the browser program runs the database data interactively through the Web server.

The B/S function is a new MIS platform based on Web technology, using a three-tier client-server system. The first-level customer is the interface between the user and the entire system. Customer applications are limited to general browsing software. The second-level Web server starts the corresponding process according to the customer's request and dynamically creates a set of HTML code, which contains the processing result and returns it to the client's browser program. The three-level database server is similar to the C/S model, which is responsible for coordinating SQL requests issued by different Web servers and managing the database.

#### 3.2.2. Choice of Operating System

Choose Windows 2000 Server as the database server operating system. Choose Windows 2000 Professional as the client operating system. Windows 2000 Server is a new operating system that integrates functional systems and network functions. It is a new generation of powerful network server systems. It has a user-friendly working environment and easy to install and maintain, includes all Windows 2000 professional functions, and provides simple and efficient network management services, such as support for DHCP server, DNS server, WINS server, WWW server, and FTP server.

#### 3.2.3. Selection of Front-End Development Tools

The front-end tools currently used for database development mainly include Power Builder, Visual Basic, and Visual C++. In contrast, Visual Basic has certain advantages in interface design, but its ability to process data is not strong. Visual C++ is powerful enough to realize any required function, but its disadvantages are the difficulty of control, the heavy workload of programming, and the long growth cycle. Power Builder has great advantages in processing large amounts of data. It is a visual development tool, which is characterized by solid code, high operating efficiency, easy to learn, easy to use, and good maintainability. It has good connections with different database systems and supports the Internet. Programming and remote client/server technology can generally perform all the functions that Visual C++ can achieve. It is one of the commonly used visual development tools at present and very suitable for the development of database application systems, considering the use of Power Builder as a front-end database development tool.

The article "Diabetes Risk Data Mining Method Based on Electronic Medical Record Analysis" was retracted in 2023. Reasons: unreliable results or conclusions; concerns about the data; concerns about the peer review; concerns about the citations.

This part of the experiment proposes that the above steps are used in the research experiment of diabetes risk data mining method based on electronic medical record analysis. The specific process is shown in Table 1.

## 4. Diabetes Risk Data Mining Method Based on Electronic Medical Record Analysis

### 4.1. Data Preprocessing Analysis

Data preprocessing is an important basic work in data science research and is of great significance to feature selection. There is no standard process for data preprocessing, and differentiated methods are usually adopted for different tasks and data set attributes. After a series of data preprocessing processes, it is determined that the final number of available data samples is 1959.

1. To understand the structure and distribution of the sample through the statistical description of index data such as age and gender, statistically sort out the age and gender distribution in the sample data and draw them into graphs, as shown in Table 2 and Figure 2.
2. It can be seen from the data in the table that, in the overall available samples after data preprocessing, there are 1020 male samples and 939 female samples, and the gender distribution is relatively even. From the perspective of age, the age range is comprehensive. There are samples in all age groups and the overall distribution meets the standard of data research. Among them, the sample data between 21 and 60 years old accounts for more than 90%, which is in line with people with diabetes, the general law of age division, and population.
3. Data integration is to merge and save different collected data for subsequent data mining work. The data of this study are stored in a MySQL relational database after preprocessing of the above steps. The data obtained in the above steps are used for correlation analysis. First, scan the database to find frequent itemsets. The minimum support is set to 15% until no frequent itemsets can be found. Then, correlation analysis is performed based on the frequent itemsets found. The result obtained is the association rule of diabetes and its complications.

The results of frequent itemsets are shown in Table 3 and Figure 3.

The correlation analysis results obtained are shown in Table 4 and Figure 4.

Diabetes is closely related to coronary heart disease, hypertension, fatty liver, chronic arterial obstructive disease, and abnormal lipid metabolism. By analyzing the first and last items on the scoreboard of the above association rules, it can be found that diabetes can easily cause high blood pressure and is also closely related to blood pressure, coronary heart disease, abnormal blood lipid metabolism, fatty liver, and various complications. According to related literature, common complications of diabetes are divided into annual and acute. Among them, chronic complications of diabetes mainly include diabetic nephropathy, cataracts and other eye diseases, heart disease, coronary heart disease, hypertension, cerebrovascular disease, and peripheral neuropathy. Acute complications mainly include diabetic ketoacidosis and lactic acidosis.

The article "Diabetes Risk Data Mining Method Based on Electronic Medical Record Analysis" was retracted in 2023. Reasons: unreliable results or conclusions; concerns about the data; concerns about the peer review; concerns about the citations.

### 4.2. Data Mining Analysis

#### 4.2.1. Experimental Results of Decision Tree Random Classification Algorithm

According to the decision tree model of the method part of this paper, the analysis node is used to evaluate the accuracy of the model.

The classification results of the training set and test set of all samples of the simple personal level model decision tree, simple clinical model decision tree, and complex clinical model decision tree are shown in Table 5 and Figure 5.

The prediction accuracy rates of the training set and test set of all samples of the simple personal level model decision tree, simple clinical model decision tree, and complex clinical model decision tree are shown in Table 6 and Figure 6.

The chart results show that the prediction accuracy of the three models is very high. The average prediction accuracy of the decision tree in this paper is 91.21%, the results of the training set and the test set are similar, and there is no overfitting in the training set. The comparison shows that the more the input variables considered, the higher the accuracy of model prediction. However, judging from the accuracy of the test set, the accuracy of simple clinical models and complex clinical models are the same, indicating that simple clinical models can provide specific guidance for doctors at different levels in clinical diagnosis and more convenient people monitor their physical state at any time.

#### 4.2.2. Analysis of the Accuracy of Random Forest Classification

Compare the performance on the random forest of the original data set, the data set with the cross-item added, and the data set after the cross feature selection. Through 4: 1 stratified sampling, the ratio of positive and negative samples in the two data sets is kept the same. The data set is divided into two parts: one is the training set and the other is the test set. We use the random forest algorithm to model the training set and test the test set. Random forest parameters are selected as follows: depth 10 and 1500 trees. In order to express the results of diabetes prediction using scores, the data set is divided into three parts: training set, test set, and validation set. The training set contains 8942 samples, the test set contains 4263 samples, and the validation set contains 3918 samples. Calculate the probability of diabetes in the test set and select the threshold; then verify the performance of the model on the test set. This paper uses sensitivity, specificity, and positive predictive value as evaluation indicators. The results are shown in Table 7.

The article "Diabetes Risk Data Mining Method Based on Electronic Medical Record Analysis" was retracted in 2023. Reasons: unreliable results or conclusions; concerns about the data; concerns about the peer review; concerns about the citations.

From the data in the table, it can be seen that 52.14% of diabetic patients can be distinguished among people whose diabetes risk probability is greater than or equal to 80%.

## 5. Conclusions

Data mining refers to the extraction of potentially useful information, knowledge, and knowledge hidden in the database and not known by people in advance and has certain research value and significance. At present, data mining is developing rapidly, involving various fields such as finance, information, insurance, and medical treatment, which has led to the interdisciplinary integration of computer technology, artificial intelligence technology, pattern recognition technology, and other fields.

In China, data mining technology in the medical field is still in a stage of vigorous development and continuous improvement. The continuous growth of medical data has brought bright industry prospects and large challenges to data mining. Hospital information covers all data resources of medical process and hospital activities, including clinical medical information and hospital management information. How to efficiently use and develop medical data has become a key link for researchers in data mining and analysis.

In this paper, there is still a lot of room for development in the data mining of diabetes risk electronic medical record data. This research is only a preliminary realization of the association rule analysis of data mining. We want to further improve the utilization efficiency of electronic medical record data; we need a deeper understanding and analysis of the characteristics of electronic medical record data and the concepts and methods of data mining technology, in order to make better use of mining technology to analyze and realize the value of electronic medical record data.

## Figures and Tables

**Figure 1:** Part of the technical process of this method.

**Figure 2:** Sample age and gender distribution.

**Figure 3:** Frequent subset analysis results.

**Figure 4:** Association analysis results.

**Figure 5:** Decision tree classification results of the three models.

**Figure 6:** The prediction results of the three models.

**Table 1:** Experimental steps in this paper.

Research experiment on data mining method of diabetes risk based on electronic medical record analysis	3.1	Design an electronic medical record data analysis system	1	Framework design
			2	Database logic design
	3.2	System platform selection	1	System structure
			2	Operating system choice
			3	Selection of front-end development tools

The article "Diabetes Risk Data Mining Method Based on Electronic Medical Record Analysis" was retracted in 2023. Reasons: unreliable results or conclusions; concerns about the data; concerns about the peer review; concerns about the citations.

**Table 2:** Sample age and gender distribution.

Generation	Gender	Quantity	Percentage (%)
20 and below	Male	13	0.66
	Female	8	0.41

21–30	Male	217	11.08
	Female	176	8.98

31–40	Male	261	13.32
	Female	257	13.12

41–50	Male	248	12.66
	Female	249	12.71

51–60	Male	175	8.93
	Female	161	8.22

61–70	Male	62	3.16
	Female	57	2.91

71–80	Male	41	2.09
	Female	22	1.12

80 and above	Male	3	0.15
	Female	9	0.46

**Table 3:** Frequent subset analysis results.

Number	Frequent subset	Support count	Support
1	Diabetes and hypertension	465	23.74
2	Diabetes and chronic arterial occlusion	372	18.99
3	Diabetes and dyslipidemia	515	26.29
4	Diabetes and fatty liver	417	21.29
5	Diabetes and coronary heart disease	439	22.41
6	Diabetes, hypertension, and coronary heart disease	581	29.66
7	Diabetes, hypertension, and dyslipidemia	704	35.94
8	Diabetes, fatty liver, and coronary heart disease	629	32.11

**Table 4:** Association analysis results.

Term			Confidence level (%)	Support (%)
1	Antecedent	Consequence		
2	Hypertension	Diabetes	13.01	31.26
3	Chronic arterial occlusion	Diabetes	26.71	13.57
4	Abnormal lipid metabolism	Diabetes	33.16	19.67
5	Diabetes	Fatty liver	47.52	35.61
6	Coronary heart disease	Diabetes	55.23	32.64
7	Hypertension and coronary heart disease	Diabetes	67.02	13.57
8	Diabetes and hypertension	Fatty liver	37.15	31.26
9	Diabetes and coronary heart disease	Fatty liver	42.24	19.67

**Table 5:** Decision tree classification results of the three models.

Actual classification	Simple personal level model		Simple clinical model		Complex clinical model	
	Not sick	Sick	Not sick	Sick	Not sick	Sick
Not sick	852	107	793	112	812	116
Sick	416	745	147	861	102	942
Total	1268	852	940	973	914	1058

**Table 6:** The prediction results of the three models.

Forecast result	Training set accuracy (%)	Test set accuracy (%)	Accuracy of all samples (%)
Simple personal level model	76.94	81.26	79.10
Simple clinical model	94.72	96.79	95.76
Complex clinical model	98.47	99.09	98.78

**Table 7:** Probability of diabetes risk.

Evaluating indicator	The probability of diabetes is more than or equal to 80 (%)
Sensitivity	72.13
Specificity	94.06
Positive predictive value	52.14

## Data Availability

No data were used to support this study.
